The article "Utilization of opium poppy seed oil for biodiesel production: A parametric characterization and statistical optimization" was retracted in 2025. Reasons: unreliable results or conclusions; concerns about the citations; concerns about the authorship.

# Utilization of opium poppy seed oil for biodiesel production: A parametric characterization and statistical optimization

**DOI:** 10.1016/j.heliyon.2024.e36851

**Published:** 2024-09-03

**Authors:** Zahara Razaq, Muhammad Imran Tousif, Sajida Noureen, Syed Ubaid Hussain, Muhammad Saleem, Fahad Mehmood Khan, Umer Shaukat, Humayun Riaz, Gokhan Zengin, Abeer Hashem, Ajay Kumar, Elsayed Fathi Abd_Allah

**Affiliations:** a Institute of Chemistry, Faculty of Chemical & Biological Sciences, The Islamia University of Bahawalpur, Punjab, Pakistan; b Department of Chemistry, Division of Science and Technology, University of Education, Lahore, Pakistan; c Department of Pharmaceutics, Faculty of Pharmacy, The Islamia University of Bahawalpur, Punjab, Pakistan; d Rashid Latif College of Pharmacy, Rashid Latif Medical Complex, Lahore, Pakistan; e Selcuk University, Science Faculty, Department of Biology, Konya, Turkey; f Botany and Microbiology Department, College of Science, King Saud University, P.O. Box. 2460, Riyadh, 11451, Saudi Arabia; g Amity Institute of Biotechnology, Amity University, Sector-125, Noida, Uttar Pradesh, 201313, India; h Plant Production Department, College of Food and Agricultural Sciences, King Saud University, P.O. Box. 2460, Riyadh, 11451, Saudi Arabia

**Keywords:** Opium poppy seed oil, Fatty acid methyl ester, Transesterification, Box-Behnken design, Biodiesel properties, GC-MS analysis

## Abstract

Consuming traditional petroleum-derived diesel fuel has long been associated with issues such as the depletion of natural energy resources. To solve these challenges, an alternate source like as biodiesel is an appealing option. Seed oils have long been recognized as an abundant and diverse source of biodiesel. In this study, poppy seed oil from the poppy (Papaver somniferum) was investigated for biodiesel production. Poppy seed biodiesel was generated and refined using acid-pretreated esterification with sulphuric acid prior to transesterification, as well as single-step alkaline catalyzed transesterification with methanol and potassium hydroxide. Finally, the percentage yield was compared. Using Statistica, the Box-Behnken design was applied to optimize process variables like time, temperature, catalyst concentration, and methanol-oil ratio to produce maximum yield. The relationship of process variables was also shown with the help of the Response Surface Methodology. A maximum yield of 94.87 % was obtained at optimized conditions, i.e., 90min reaction time, 60 °C of temperature, 0.25 mg of catalyst concentration, and 3v/v% alcohol-oil ratio. The fuel properties of biodiesel produced, such as acid value, moisture content, saponification value, iodine value, specific gravity, percentage of free fatty acids, refractive index, viscosity, boiling point, and peroxide value, were measured and compared with the American Society for Testing and Materials (ASTM) D6751 and European Standards (EN) 14214. Further results were studied and discussed using Fourier Transfer Infrared (FTIR) analysis, which showed maximum similarity of raw material to formed biodiesel. Gas Chromatography-Mass Spectrometry (GC-MS) analysis was performed to identify and quantify various fatty acid methyl esters. The results obtained were in accordance with various international standards for biodiesel fuel. Thus, poppy seeds can be used to obtain biodiesel.

## 1 Introduction

Energy resources like fossil fuels are limited and non-renewable, but the demand for these resources is increasing rapidly [[1], [2], [3]]. “It will take less than ten decades for fossil fuel reserves to be depleted,” the prediction by the World Energy Forum. Thus, there is an imperative need to find an alternative source for this vital form of energy, especially in sectors like industrialization and transportation [[4], [5], [6], [7]]. Biofuels are very appealing in replacing traditional fuel and can reduce the energy crisis. Among various types of biofuels, biodiesel is becoming more accepted because of its properties and chemical nature. It is worth mentioning that no engine modification is required when using biodiesel as fuel [8]. Biodiesel (BD) is composed of fatty acid methyl esters (FAME) (C16-C18) obtained through transesterification process [[9], [10], [11]]. Comprehensively described, BD is a mixture of esters (usually monoalkyl, methyl, or ethyl) of fatty acids when renewable biological resources, such as plant oils or animal fats containing triacylglycerides (TAGs), undergo transesterification. In the transesterification reaction three molecules of fatty acids ester and one molecule of glycerin are obtained from one molecule of TAG [12]. Various factors including physical properties, chemical composition, oil content, and lastly, suitability, are considered in the selection of feedstock [13]. Primary feedstock classification includes edible oil, non-edible oil, recycled or waste oil, and animal fats. Biofuel from algae has also been experimented and utilized as a source [9,14,15].

Vegetable oils include edible and nonedible oils. Edible oils are produced in many areas geographically, thus serving as the primary feedstock, and noticeable properties of biodiesel from edible oil are suitable to substitute diesel fuel. However, excessive use of edible oil as feedstock can be a possible cause of competition and an increase in the biodiesel cost from this source [[16], [17], [18]]. Opium poppy (*Papaver somniferum*) belongs to the family Papaveraceae subfamily Papaveroideae. Famous Unani scholar Avicenna stated that various poppy seed varieties include wild, garden, black, and horned poppy. Poppy seeds are primarily white and black. While [19] we studied three poppy seed varieties (white, yellow, and blue). The production of biodiesel using various methods depends on the feedstock's type and nature. These techniques and processes include transesterification. Catalytic distillation, reactive distillation, thermal cracking or pyrolysis, micro-emulsion, and supercritical fluid techniques, while *transesterification* is a very common, simple, and widely used technique [13,[20], [21], [22]]. The current project focusses on the production, optimization, and characterization of biodiesel derived from poppy seed using the transesterification method, Box-Behnken Design for yield optimization, and a variety of characterization techniques.

## 2 Experimental

### 2.1 Feedstock

Opium poppy seeds were purchased from the local market of Bahawalpur, Pakistan. Seeds were heated and pressed mechanically to obtain oil, and later purification was achieved initially through layered cotton cloth [23] and filter paper [24]. Finally, a cotton plug passed oil through the funnel [25]. Two-step esterification and single-step transesterification techniques were used to obtain and compare FAME yield.

### 2.2 Biodiesel production

The following processes were employed to obtain biodiesel.

i. Single Step Transesterification (Base Catalyzed)
ii. Two Two-step esterification (Acid catalyzed/Pre-Treatment)

#### 2.2.1 Single-step transesterification (base catalyzed)

A single-step process (Fig A.1) where the oil (50 ml) was heated (50 °C) for a specific time (1–2 min). Then, 2 g of potassium hydroxide as a catalyst was dissolved in 18 ml of methanol in a 250 ml round bottom flask containing a magnetic stirrer. Then, pre-heated oil was gently poured into it. This reaction mixture was stirred for 75 min with maximum rpm speed at 60 °C [24]. This round bottom flask was attached with a reflux condenser set carefully so that methanol would not be evaporated if the reaction temperature accidently rose higher than 60 °C [26]. The mixture was then transferred into a 250 ml separating funnel. Glycerol and formed biodiesel layers appeared immediately while the separation funnel was allowed to stand for at least 24 h or left overnight to obtain a fine separation. After the specified time, glycerol was drained from the separating funnel, and the methyl ester was washed with pre-heated distilled water (100 °C) until it became clear. It was done to remove excess amounts of methanol and impurities. Methyl ester was then allowed to heat at 60 °C until clear biodiesel was obtained [27]. The yield was calculated using Equation (1).

Eq. 1 $$\text{Biodiesel}\;\text{Yield}\;\left(\%\right)=\frac{Weight\;of\;fattyacid\;methylester}{weight\;of\;oil\;used}\times 100\%$$

#### 2.2.2 Two-step transesterification (acid catalyzed/pre-treatment)

In this method, initially, 10 ml of 5 % H_2_SO_4_ solution as a catalyst was added to 20 ml methanol. This acid treatment was performed as a pretreatment to decrease the free fatty acid value (<2 %). Then, 50 ml of preheated poppy oil was added. Heat at stir at 60 °C at maximum speed on a magnetic stirrer hot plate. Put this in a separating funnel. Two layers were formed. Taking the lower oil layer for the next step, the upper methanol layer was wasted. The obtained oil was subjected to base catalyst transesterification as described in the earlier single-step method.

### 2.3 Statistical design and optimization

To optimize reaction conditions, Box-Behnken experimental (BBD) design with 3 blocks and 4 factors (3^2^ × 4–1), including 27 experiments, was applied using TIBCO Statistica Software (version 13.5.0). The levels and range values are shown in Table A.1. The BBD is chosen for its efficient experimentation, which reduces the number of experiments and provides intermediate benefits. It enables a three-level design and identifies optimal conditions for maximizing biodiesel yield or quality through efficiently navigating the experimental area and determining the parameters that produce the best reaction [28].

A total of 27 experiments were carried out randomly to avoid systemic error. The effects of four independent variables—time, temperature, catalyst concentration, and alcohol: oil ratio—were studied to optimize the dependent variable output. First-order and Second-order polynomial models were constructed, and response surface methodology was used to relate the response of independent and dependent variables.

### 2.4 Physiochemical properties evaluation

The physicochemical characteristics of oil and biodiesel were determined and compared to international standards ASTM D6751 and EN 14214 [29].

#### 2.4.1 Determination of the moisture content

Analytically weighed 2 g of sample was placed in an oven at 100 °C. After every 30 min the sample was taken out, cooled, and weighed. This procedure was repeated until a constant weight was obtained [27]. The percentage moisture content (% wt.) was calculated according to Eq. 2

Eq. 2 $$\text{Percentage}\;\text{moisture}\;\text{content}=\frac{{W_{1}-W}_{2\;}}{W_{1}}\times 100$$

where, *W*_*1*_ = original weight of the sample before drying, *W*_*2*_ = weight of the sample after drying.

#### 2.4.2 Determination of saponification value

Accurately weighed, 1 g of each sample was dissolved in 25 ml of 0.5 M ethanolic potassium hydroxide solution. This flask was heated under reflux for almost 30 min with occasional stirring. This resultant solution was titrated with 0.5 M HCl solution using phenolphthalein indicator [27]. The saponification value, SV (mg KOH), was calculated using the following equation Eq. 3

Eq.3 $$\text{Saponification}\;\text{value}=\frac{56.1\times M\times \left(B-V\right)}{W}$$

where, *M* = molarity of standard HCl, *B* = volume of HCl used in blank titration, *V* = volume of HCl added, 56.1 = molar mass of potassium hydroxide, and *W* = weight in gm of sample.

#### 2.4.3 Determination of iodine value

About (0.10–0.15 g) of each sample was weighed and transferred to a 500 ml flask. 15 ml of 96 % ethanol was dissolved in that flask while stirring for 5 min. Later, 20 ml of 0.1 mol/L ethanolic iodine solution was added. Stirring continued for a few minutes and slowed down to add 200 ml of distilled water (cold). Finally, after 5 min of stirring, the resultant solution was titrated with standardized sodium thiosulphate using a starch indicator.

Eq.4 $$\text{Iodine}\;\text{Number}=\frac{\left(B-A\right)\times C\times 12.69}{m}$$

where, B = Volume (mL) of sodium thiosulfate solution used for blank titration; A = Volume (mL) of sodium thiosulfate solution used for sample titration; C = Concentration (mol/L) of the sodium thiosulfate solution and m = aliquot weight (gm).

#### 2.4.4 Determination of acid value

The sample was weighed (1 g) and dissolved in a neutral mixture of absolute alcohol (12.5 ml) and diethyl ether (12.5 ml), resulting in an oil solution which was titrated using 0.1 M potassium hydroxide solution using phenolphthalein as an indicator. Equation Eq. (5) was used to find the acid value (mg KOH/g)

Eq. 5 $$\text{Acid}\;\text{value}=\frac{56.1\times M\times V}{W}$$

where, *M* = molarity of standard KOH (0.1 M), *V* = volume (ml) of KOH, 56.1 = molar mass of potassium hydroxide, and *W* = weight (gm) of sample.

#### 2.4.5 Determination of free fatty acid (FFA)

Each sample equivalent to 1 g was dissolved in a neutral mixture of absolute alcohol (12.5 ml) and diethyl ether (12.5 ml). The resultant oil solution was titrated using 0.1 M potassium hydroxide solution using phenolphthalein as an indicator. Following equation Eq. (6) was used to find the acid value

Eq. 6 $$\text{FFA}\;\left(\%\right)=\frac{0.0282\times TV\times 100}{W}$$

where, 0.0282 (constant) = weight of oleic acid neutralized by KOH (1 mg); *TV =* titer value and *W* = weight (gm) of sample.

#### 2.4.6 Determination of ester value

The ester value for seed oil and product was calculated through the difference between the saponification and acid values. So,

Eq.7 Estervalue=Saponificationvalue‐Acidvalue

#### 2.4.7 Determination of peroxide value

Accurately weighed 1 g of potassium iodide was taken in a test tube and solvent mixture containing 2 ml of glacial acetic acid and 1 ml of chloroform was added. Then 1 g of each sample oil was added respectively in each tube. The tube was then allowed to boil for 30 s in boiling water. All the boiling tubes poured into these flasks filled with 20 ml of 5 % potassium iodide solution. Then, they were allowed to titrate with sodium thiosulphate (0.002M) using a starch indicator until the yellow color disappeared. A blank (without sample) was also run in the same way under the same conditions [27]. The peroxide value was checked by the following equation Eq. (8).

Eq. 8 $$\text{Peroxide}\;\text{value}\;\left(\text{millieq}/\;100g\;\text{sample}\right)=\frac{\;N\times \left(V-B\right)\times 1000}{W}$$

where, N = normality of sodium thiosulphate solution, *B* = titration of blank in ml, *V* = titration of test sample in ml, *W* = weight of the sample, and 1000 = standard factor of peroxide value.

#### 2.4.8 Determination of viscosity

Viscosity was measured with a viscometer (Brookfield) using a spindle. The temperature of the magnetic hot plate was constant while the temperature of samples was elevated to different values.

#### 2.4.9 Determination of refractive index

Each sample (1–2 drops) was put on the glass slide of the refractometer (ATAGO RX 5000α). All the samples were checked at the same time and temperature. Hence, the refractive index of all samples was determined.

#### 2.4.10 Determination of boiling point

A hotplate was used for this purpose. 20 ml of each sample was taken in a beaker. A thermometer was carefully inserted in each beaker and fully covered when placed on a hot plate. As the temperature rises, the point at which the sample started boiling, was noted. This was the boiling point.

#### 2.4.11 Determination of cloud and pour point

The cloud point of every sample was checked by taking 20 ml of each sample in a beaker and keeping all beakers one by one in the freezing zone of a 1000 ml beaker containing a mixture of ice and salt until clouds of crystal appeared at the bottom. For the pour point, 20 ml of each sample was poured into a 50 ml beaker. They were kept in the refrigerator to solidify. When the beaker was brought out in an open place, the temperature was noted when it melted and started flowing.

#### 2.4.12 Average molecular weight (MW) determination

The average molecular weight (MW) of the samples was calculated based on the saponification value (SV) and the acid value (AV) of the samples using the following formulae in Equation (9) [30].

Eq.9 $$\text{MW}\;\left(g/\text{mol}\right)=\frac{\;56.1\times 1000\times 3}{\left(SV-AV\right)}$$

#### 2.4.13 Cetane number and higher heating value

The cetane number (CN) and higher heating value (HHV) of the samples were calculated based on the saponification value (SV) and the iodine value (IV) of the samples using the following formulae in Equations. Eq.10, Eq.11), respectively [31].

Eq.10 $$\text{CN}=46.3+\frac{5458}{\text{SV}}\;‐0.225\times \text{IV}$$

Eq.11 HHV=49.43−[0.041(SV)+0.015(IV)]

### 2.5 FTIR analysis

A FTIR (Bruker, Germany) spectrophotometer was used to obtain spectral information on functional groups present in all samples. It was performed by placing a small drop of liquid sample on a KBr pellet. All the spectra were recorded within the wavenumber range of 4000 to 700 cm^−1^ with a resolution of 4 cm^−1^, and 12 scans were averaged to obtain a final spectrum.

### 2.6 GC-MS analysis

GC-MS was used to analyze the composition of the product. The oven temperature of GC was held at the initial temperature of 60°C for 2 min, then ramped to a final temperature of 250°C at a rate of 15°C/min, held for 5 min, and then ramped to a final temperature of 320°C at a rate of 10°C/min, held for 2 min with a total run time of 32.7 min.

## 3 Results and discussion

### 3.1 Yield

For alkali-treated biodiesel, the highest yield obtained was 94.87 % with; 90 min (time), 60 °C (temperature), 0.25 mg (catalyst concentration), and 3v/v% (alcohol-oil ratio). The maximum yield obtained for acid-treated biodiesel was 91.21 % at 10 v/v% methanol to oil ratio, 1.25 g KOH catalyst, and 40 °C in 90 min as stated in Table B.1.

### 3.2 Optimization of transesterification

Predicted and experimental percentage of the biodiesel yield from poppy seed for design matrix of variables and BBD is shown in Table B.2 with *p*-values in Table B.3. Furthermore, the plot of Experimental against Predicted values is given in Fig. B.1.

Fig. B. 2 shows profiles of predicted values and desirability, which indicates the individual response of each process parameter on desirability, i.e., yield. From the graphs in Fig. B.3, reaction time is directly related to yield, while the optimum values for temperature, catalyst concentration, and alcohol-oil ratio are 60 °C, 0.75 mg, and 6.5 v/v, respectively. These parameters may have a varying negative effect on yield.

Equation 12 Output(%)=7.30500(Time)−3.68056(Temp)+0.26556(Cat.Conc)+3.72389(Al−OilRatio)+72.85296

Equation 13 Output(%)=7.30500(Time)−3.68056(Temp)+0.26556(Cat.Conc)+3.72389(Al−OilRatio)+1.98778(Time×Temp)−2.39844(Time×Cat.Conc)−4.48156(Time×Al−OilRatio)−0.81378(Temp×Cat.Conc)−1.84711(Temp×Al−OilRatio)+1.58111(Cat.Conc×Al−OilRatio)+72.85296

Table B.3 depicts coefficient and p-value values. The values indicate that time, temperature, and the Alcohol: oil ratio significantly affect the percentage yield obtained. The p-value (0.000064) obtained from time indicates that time has a greater impact on percentage yield.

### 3.3 Response surface methodology (RSM)

RSM allowed us to study the effect of independent variables providing three-dimensional response surface graphs. Consequently, several response surface graphs representing the effects of these independents during transesterification are shown in Fig. B.3. After the study of these graphs, optimum conditions for the maximum yield were determined. The results indicated that for specific combinations different variables have different effects on the output of biodiesel. When the alcohol-oil ratio and catalyst concentration were seen in the response surface (Fig B.3i). Increasing both variables had a positive effect on the yield (%). When studying the alcohol: oil ratio with temperature increasing the ratio while decreasing the temperature provides maximum yield (%) as in Fig B.3ii. Catalyst concentration and temperature are inversely related when output percentage yield is considered (Fig B.3.iii). The combined response surface graph for time and temperature showed that less time needed more temperature to produce maximum biodiesel (Fig B.3iv). The effect of alcohol: oil ratio with time showed similar effects when alcohol: oil ratio with catalyst concentration (Fig B.3v). Increasing collectively the alcohol: oil ratio and time will increase output. When studying the effect of catalyst concentration for the effect of time on yield graph showed that less catalyst concentration requires more time (Fig B.3vi).

### 3.4 Biodiesel physicochemical properties

Physicochemical properties of produced biodiesel (PBD) and pretreated biodiesel (PPBD) were in good agreement with American and European standards and summarized in Table B.4. In a study where waste frying oil was used to obtain biodiesel (WFBD), physicochemical properties were only compared to European standard, the acid value (0.428m KOH/g), moisture content (0.035%Wt) and density (0.87 g/cm^3^) values were calculated and found are comparable to our results. However, the WFBD has a lower saponification value (194 mg KOH/g oil) and a greater pour point (11°C) than PBD and PPBD [32]. Higher saponification values indicated that more alkali is required to convert poppy seed oil to biodiesel, and a lower pour point is desirable so that biodiesel can retain its flow properties at very low temperatures. Only temperature-related properties were studied in a study where Karanja and Jatropha oils were used to produce plant-scale biodiesel. Viscosity (mm^2^/sec) of 5.18 and 4.53 were obtained with pure biodiesel from Karanja and Jatropha oil, respectively. It is higher than the obtained viscosity from PBD and PPBD. Both values are near the upper limit set by international standards, i.e., ASTM D6751 and EN 14214 [33].

### 3.5 FTIR spectroscopy

FTIR analysis was evaluated to assess the completion of the transesterification reaction and the conversion of poppy seed oil into fatty acid methyl esters. Only a slight difference can be noted in all spectra that signifies that obtained biodiesel is almost similar to their starting materials (oils), as shown in Fig B.4. In all spectra, bands are present in the region of 2800–3000 cm^−1^ that may be due to symmetric CH_2_ and asymmetric CH_3_ and CH_2_ stretching. In the 1800-1700 cm^-1^ region, bands are present, resulting in C=O stretching. This band is also present in all samples. CH_3_ asymmetric bending and methyl ester deformation vibration at 1435.56 cm^−1^ were observed in FTIR spectra of biodiesel. These bands appeared at 1461.40 cm^−1^ for biodiesel obtained after pretreatment. These bands are not present in the FTIR spectra of poppy seed. Moreover, in FTIR spectra of biodiesel, O-CH_3_ stretching was observed at 1169.33 cm^−1^ in biodiesel and 1159.46 cm^−1^ in pretreated biodiesel. The glycerol group band was seen at 1377.26 cm^−1^ in the FTIR spectrum of poppy-seed oil, which was absent in the biodiesel spectrum. The existence of regions of 1741.20 cm^−1^, 1741.31 cm^−1,^ and 1743.32 cm^−1^ in FTIR spectra of poppy seed and both biodiesels, respectively, showed C-H stretching. These findings were in accordance with previous work [34].

FTIR spectra of all samples showed strong intensities of asymmetric stretching vibration for = C-H at 2924 cm^−1^ while symmetric stretching vibrations band for -CH_2_ was seen at 2854 cm^−1^. C=O stretching was observed at 1738-1743 cm^-1^ for these various samples. In another work, FTIR spectrum of methyl esters showed absorbance at the same wavenumbers for = C-H and -CH_2_ while –C=O stretching was seen at 1742.1 cm^−1^ [35]. Another study, where a mixture of edible line seed oil, and palm oil with non-edible oils was used to produce biodiesel, supported our findings as a region of 2800–3000 cm^−1^ and 1675–1725 cm^-1^ represented the CH_3_ stretching vibration and the stretching of carbonyl group respectively [36].

### 3.6 GC-MS analysis

GC-MS analysis of the both poppy seed oil and biodiesel were done as shown in Fig. B 5 and 6. It can be seen that the biodiesel (PBD) obtained primarily contained three fatty acid methyl esters and others were present in minor quantities, as mentioned in Table B.5. The GC-MS analysis indicated that the key ethyl esters were of as of Octadecadienoic acid and Hexadecanoic acid and highest percentage was of 9,12-octadecadienoic acid (Z, Z)-methyl ester. The formation of methyl esters is due to the production of high methoxide radicals during the reaction [37]. The composition of biodiesel produced differs from conventional diesel fuel, which mainly consists of n-alkanes, iso-alkanes, and cyclo-alkanes [29]. In another study, it was demonstrated that diesel is a complex mixture of hydrocarbons (C_8_-C_40_). Three different samples of diesel fuel were analyzed with the GC-MS analysis technique, and the key methyl ester found was linolenic acid methyl ester.

### 3.7 Analysis of diesel and components via GC-MS

The different composition is due to divergent feedstock origin and chemical structure, as biodiesel feedstock are predominantly composed of triglycerides and free fatty acids, which undergo chemical reactions to yield FAMEs, the primary components of biodiesel. However, conventional diesel fuel is derived from crude oil, a fossil fuel composed mainly of hydrocarbons, while biodiesel is dominated by the ester functional group [4,38].

### 3.8 Challenges

The main obstacle to producing biodiesel from vegetable oils is the feedstock, which could increase costs [39]. Loss of biodiversity, deforestation, and ecosystem changes are other challenges in biodiesel scale-up production [40]. Other potential issues include inefficient procedures and altered fuel characteristics that affect engine performance [38,41].

### 3.9 Conclusion and future prospective

The study investigated biodiesel production from poppy seed via transesterification and esterification processes, utilizing methanol and KOH as a catalyst under controlled temperature and time conditions. The biodiesel production from opium poppy seed achieved a maximum yield of 94.87 %. The model demonstrated that variables such as time, temperature, and the alcohol-to-oil ratio significantly influenced the biodiesel yield. Following production, the quality parameters of the biodiesel were evaluated according to ASTM D6751 and EN 14214 standards. FTIR analysis confirmed the biodiesel's stability, while GC-MS results revealed that 12-octadecadienoic acid (Z, Z)-methyl ester was present in the highest concentration. Producing biodiesel from vegetable oils offers a more environmentally sustainable alternative to fossil fuels. Compared to conventional diesel, biodiesel can significantly reduce emissions of greenhouse gases, particulate matter, and other pollutants. Future research will focus on studying the blends of poppy seed for their physicochemical properties, thermal behavior, fatty acid profile, and engine performance. Economic analyses of biodiesel production are essential for identifying practical strategies to enhance output, such as optimizing feedstock logistics and supply chains. Comparative studies will be conducted using different feedstock processing techniques and catalysts to assess biodiesel production from poppy seed. Engineering research will address technical challenges, including improving biodiesel's cold flow properties and oxidative stability, to ensure it meets performance standards for diesel engine applications. Further investigation is needed to understand the impacts of biodiesel production on communities, particularly concerning land use changes and food security issues related to feedstock cultivation.

## Funding

The authors would like to extend their sincere appreciation to the Researchers Supporting Project Number (RSP2024R134), King Saud University, Riyadh, Saudi Arabia.

## Author contributions

Conceptualization: S.N. and S. U.H.; methodology, data collection and original data analysis: Z.R., F.M.K., U.S. and H.R; data presentation, writing: M.S. and M.I.T; reviewing and editing: A.H., A.K. and E.F.A.; funding acquisition: A.H. and E.F.A.

## Declaration of competing interest

The authors declare that they have no known competing financial interests or personal relationships that could have appeared to influence the work reported in this paper.

I, **Muhammad Imran Tousif** on behalf of all co-authors submits the declaration of interests that there are no Competing interests for this manuscript.

## Figures and Tables

**Table A.1:** Independent variables and levels used for study design.

Code	Independent Variable	Unit	Factor Levels		
			−1	0	+1
X_1_	Time	min	15	52.5	90
X_2_	Temperature	^o^C	40	60	80
X_3_	Catalyst Concentration	mg	0.25	0.75	1.25
X_4_	Alcohol: Oil Ratio	(v/v)	3	6.5	10

**Table B.1:** Percentage yield of all biodiesel, pretreated biodiesel and blends (B1-B5).

Product	Yield (%)
Biodiesel	94.87
Pretreated Biodiesel	91.21

**Table B.2:** Experimental percentage yield as output for biodiesel production from poppy seed oil.

Run Order	Time (min) X_1_		Temperature (^o^C) X_2_		Catalyst Concentration (mg) X_3_		Alcohol: Oil Ratio (v/v) X_4_		Yield (%) Output	
	Coded	Real	Coded	Real	Coded	Real	Coded	Real	Experimental	Predicted
1	−1	15	−1	40	−1	0.25	−1	3	60.77	60.77
2	−1	15	−1	40	0	0.75	+1	10	80.98	79.33
3	−1	15	−1	40	+1	1.25	0	7	69.97	71.56
4	−1	15	0	60	−1	0.25	+1	10	73.87	74.97
5	−1	15	0	60	0	0.75	0	7	75.15	67.82
6	−1	15	0	60	+1	1.25	−1	3	60.78	63.89
7	−1	15	+1	80	−1	0.25	0	7	53.88	54.89
8	−1	15	+1	80	0	0.75	−1	3	52.88	51.59
9	−1	15	+1	80	+1	1.25	0	10	67.71	71.17
10	0	52.5	−1	40	−1	0.25	+1	10	75.85	78.93
11	0	52.5	−1	40	0	0.75	0	7	66.34	71.19
12	0	52.5	−1	40	+1	1.25	−1	3	71.75	82.10
13	0	52.5	0	60	−1	0.25	0	7	77.77	74.65
14	0	52.5	0	60	0	0.75	−1	3	67.99	70.76
15	0	52.5	0	60	+1	1.25	0	10	80.78	81.87
16	0	52.5	+1	80	−1	0.25	−1	3	61.25	65.65
17	0	52.5	+1	80	0	0.75	+1	10	71.35	67.09
18	0	52.5	+1	80	+1	1.25	0	7	70.48	66.72
19	0	90	−1	40	−1	0.25	0	7	85.35	83.29
20	0	90	−1	40	0	0.75	−1	3	75.45	78.83
21	+1	90	−1	40	+1	1.25	0	10	85.57	81.45
22	+1	90	0	60	−1	0.25	−1	3	94.87	90.09
23	+1	90	0	60	0	0.75	+1	10	82.13	83.06
24	+1	90	0	60	+1	1.25	0	7	75.88	82.11
25	+1	90	+1	80	−1	0.25	+1	10	75.11	75.47
26	+1	90	+1	80	0	0.75	0	7	72.54	75.14
27	+1	90	+1	80	+1	1.25	−1	3	80.58	78.05

**Table B.3:** Significance of individual parameters and 2-way interactions.

Parameter	Coefficient	p-Value
1.Time	7.30500	0.000064∗
2.Temp	−3.68056	0.010758∗
3.Catl. Conc	0.26944	0.831434
4.Alcohol-Oil Ratio	3.72389	0.010071∗
1∗2	1.98778	0.222231
1∗3	−2.39844	0.146299
1∗4	−4.48156	0.013264∗
2∗3	0.81378	0.607765
2∗4	−1.84711	0.254683
3∗4	1.58111	0.326027

∗p < 0.05 = significant values.

**Table B.4:** Physicochemical properties of biodiesel and pretreated biodiesel.

Properties	PO	PBD	PPBD	ASTM D6751	EN 14214
Acid Value (mg KOH/g)	1.32	0.39	0.42	Max 0.5	Max 0.5
Moisture Content (% Wt.)	1.375	0.034	0.037	Max 0.05 %	–
Saponification Value (mg KOH/g oil)	204.33	254.68	252.23	–	–
Iodine Value (gI_2_/100 g oil)	128.58	61.69	68.15	–	Max 120
Specific Gravity	0.96	0.86	0.85	0.86–0.90	0.85
Cloud Point (°C)	12.4	1.6	1.3	−3 to 12	–
Pour Point (°C)	7.4	−1.2	−1.5	−15 to 16	–
Free Fatty Acid (%)	0.89	0.18	0.21	–	–
Refractive Index at 20°C	1.470	1.453	1.385	–	–
Viscosity at 40°C (mm^2^/s)	25.96	4.18	4.24	1.9–6.0	3.5–5.0
Boiling Point (°C)	320	260	258	–	–
Peroxide Value (meqO_2_/kg)	3	28	26	–	–
Density (g/cm^3^)	0.92	0.89	0.89	0.88	0.86–0.90
Cetane Number	44.08	53.85	52.61	Min. 47	Min. 51
Average Molecular Weight (g/mol)	829.02	661.84	668.36	–	–
Higher Heating Value (M.Jkg^−1^)	39.12	38.06	38.07	–	–

**Table B.5:** GC-MS analysis of poppy seed oil and obtained biodiesel.

Compounds detected	R_t_ (Retention Time)		Percentage	
	Poppy seed Oil	Biodiesel	Poppy seed Oil	Biodiesel
Octanoic acid, methyl ester	–	6.519	–	0.24
Dodecanoic acid, methyl ester	–	10.315	–	0.27
9-Hexadecenoic acid, methyl ester,	–	13.162	–	2.33
Hexadecanoic acid, methyl ester	13.283	13.313	2.45	11.66
Ecgonine Methyl Ester	–	13.747	–	4.61
11-Octadecenoic acid, methyl ester	14.424	–	3.98	–
9,12-Octadecadienoic acid (Z,Z)- Methyl Ester	–	14.797	–	15.04
9-Octadecenoic acid (Z)-, Methyl Ester	–	15.009	–	9.32
Tetracosanoic acid, methyl ester	–	21.066	–	1.42
Pentacosanoic acid, methyl ester	–	22.288	–	0.27
Hexacosanoic acid, methyl ester	–	23.368	–	0.40

**Fig. A.1:** Single step transesterification.

**Fig. B.1:** Predicted yield (%) versus experimental yield (%) plot.

**Fig. B.2:** Predicted values and desirability.

**Fig. B.3:** Response surface graphs of biodiesel output (%) at various (A) alcohol: oil ratios and catalyst concentrations, (B) alcohol: oil ratios and temperatures, (C) catalyst concentrations and temperatures, (D) times and temperatures, (E) alcohol: oil ratios and times, and (F) catalyst concentration and times.

**Fig. B.4:** FTIR of (a) opium poppy oil and (b) biodiesel from opium poppy oil (c) acid treated biodiesel.

**Fig. B. 5:** Total ion chromatogram of poppy seeds oil.

**Fig. B. 6:** Total ion chromatogram of biodiesel.
